This article has been retracted.

# Pathological stage-associated non-coding RNA long intergenic non-protein coding RNA 1234 (LINC01234) participation in cell cycle regulation in adrenocortical carcinoma through bromodomain-containing protein 4 (BRD4) expression mediation via sponging microRNA (miR)-140-3p

**DOI:** 10.1080/21655979.2022.2081464

**Published:** 2022-06-29

**Authors:** Dan-Dan Zhu, Xin-Bo Yu, Wen Jiang, Yu Zhu

**Affiliations:** Department of Urology, Ruijin Hospital, Shanghai Jiao Tong University School of Medicine, Huangpu, Shanghai, China

**Keywords:** LINC01234, ACC, cell cycle, BRD4, miR-140-3p

## Abstract

Many researches indicated that long non-coding RNAs (lncRNAs) were involved in the malignant progression of tumors, including Adrenocortical Carcinoma (ACC). However, as for most lncRNAs, their biological behaviors and molecular mechanism remain unclear in ACC. In the present research, weighted gene co-expression network analysis (WGCNA) was used to identify pathologically relevant gene, including lncRNAs. By comparing their expressions in GSE61359 tumors and normal controls, long intergenic non-protein coding RNA 1234 (LINC01234) was selected to investigate the clinical significance, biological function, and mechanism in ACC. Data mining revealed that LINC01234 expression was significantly up-regulated in ACC patients, and a shorter survival time presents in patients with higher LINC01234 expression compared to that in patients with lower LINC01234 expression. Further, LINC01234 silencing resulted in cells growth arrest in vitro and in vivo. Mechanism studies suggested that LINC01234 silencing induced cell cycle arrest, and bromodomain-containing protein 4 (BRD4) overexpression could restore this phenomenon. Further research showed that LINC01234 could mediate BRD4 expression through competitively sequestering microRNA (miR)-140-3p, as evidenced by the positive correlation of LINC01234 with BRD4 and inverse correlation with miR-140-3p expression. Luciferase activity assay also verified the targeting relationship between LINC01234, BRD4 and miR-140-3p. And up-regulated LINC01234 in ACC cells significantly reversed the degradation of BRD4 by miR-140-3p. Collectively, we deduce that LINC01234 functions as a ceRNA to regulate BRD4 expression by sponging miR-140-3p in ACC progress. Our findings have the potential to provide a new target for the diagnosis and treatment of ACC.

## Highlights

- LINC01234 is a novel pathological–associated lncRNA.
- Upregulated LINC01234 means worse prognosis in ACC.
- LINC01234 silencing induces cell cycle arrest.
- LINC01234/ miR-140-3p /BRD4 axis is involved in cell cycle in ACC.

## Introduction

Adrenocortical carcinoma (ACC) is a rare malignancy which hardly shows any obvious clinical symptoms in the early stage [1,2]. Even more serious, conventional radical surgery has little effect on patients with advanced metastases [3]. For patients undergoing surgical treatment, the probability of recurrence is high, which leads to a poor prognosis [4]. At present, no clear molecular markers have been confirmed for early ACC progression. Moreover, the specific molecular mechanism of ACC is still not fully elucidated. Hence, it is critical to explore diagnostic markers related to the progress of ACC and to investigate novel effective treatments.

Weighted gene co-expression network analysis (WGCNA) is a bioinformatic method that can be performed to explore relationships between high throughput data and sample characteristics [5]. WGCNA has been applied to identify novel long non-coding RNA (lncRNA) biomarkers of tumors and to identify abundant lncRNAs associated with tumor prognosis [6,7]. To date, WGCNA has not been used for the identification of lncRNAs in ACC. The prognoses of patients with ACC with various pathological stages are vastly different [8]. Hence, WGCNA was used in this study to explore relationships between lncRNAs and pathological stages.

LncRNAs, a set of RNAs with less than 200 nucleotides and no coding capacity, have emerged as a novel research focus in tumorigenesis [9]. In recent years, accumulating evidence has linked dysregulation of lncRNAs with malignant tumor progression through multiple biological processes, including chromatin modification [10], X-chromosome inactivation [11], microRNA (miRNA) sponging [12], etc. LINC01234, located at 12q24.13, is a highly abundant, conserved mammalian non-coding RNA. Initially, LINC01234 was universally known for its participation in predicting the survival rate of breast cancer [13]. In hepatocellular carcinoma (HCC), LINC01234 was involved in proliferation and chemoresistance through the MAGEA3/LINC01234/miR-31-5p axis [14]. In colon cancer, LINC01234 competitively binds miR-642a-5p to promote serine hydroxymethyltransferase 2 expression for accelerating cell proliferation [15]. However, few studies have been carried out to clarify the biological function of LINC01234 in the progression of ACC.

In this study, LINC01234 was first identified as a novel pathological-associated lncRNA and its role in ACC was discovered. And data mining revealed that markedly up-regulated LINC01234 was observed in ACC, suggesting a poor prognosis. Hence, we hypothesized that LINC01234 plays a pro-tumor role in tumor progression. And the Assay results confirmed this hypothesis.

## Materials and methods data mining

In this study, The Cancer Genome Atlas (TCGA) and two Gene Expression Omnibus (GEO) datasets (GSE61359 and GSE33371) were used to analyze lncRNA expression patterns in ACC. The GEO data can be found at https://www.ncbi.nlm.nih.gov/geo. In addition, the Gene Expression Profiling Interactive Analysis (GEPIA) database was used (http://gepia2.cancer-pku.cn/) to uncover the prognostic significance of LINC01234 and BRD4 in TCGA-ACC.

### RNA-Seq data preprocessing and co-expression network construction

RNA-Seq matrices with corresponding clinical information were downloaded from TCGA-ACC, and then data standardization was performed by transforming the reads per kilobase per million mapped reads (RPKM) of genes into transcripts per kilobase of exon model per million mapped reads (TPM). A total of 60,483 genes from 79 ACC samples were annotated as gene symbols and biotypes using version 22 of the GENCODE annotation file, and 34,185 genes belonging to messenger RNAs (mRNA) and lncRNAs were separated from the matrix table. Genes with quartile values of TPM <0.3 were discarded, and the remaining abundantly expressed genes (AEGs) were reserved. To narrow the very large span of TPM, they were then converted into the log2 form (TPM + 1) for subsequent analysis.

WGCNA was performed to identify pathologically relevant lncRNAs as previously described [5]. First, the AEG expression matrix of ACC samples was evaluated to select suitable samples and genes. Then, a scale-free co-expression network for the AEGs was constructed using the WGCNA R package [5]. The distance among ACC samples was evaluated by average linkage clustering, and the reliability of network construction was ensured by removing the outlier samples. A suitable soft-thresholding parameter β was chosen to ensure network construction in accordance with the characteristics of the scale-free network. The adjacency matrix was transformed into a topological overlap matrix (TOM) to measure the network connectivity of a gene, as well as to calculate the corresponding dissimilarity (1-TOM). According to the TOM-based dissimilarity measure, average linkage hierarchical clustering was performed to conduct a gene dendrogram (minimum size of module = 30). Some modules for the subsequent analysis were merged by calculating the dissimilarity of module eigengenes (MEs).

### Cell culture

SW-13 and H295R cells were purchased from ATCC (Manassas). DMEM (Solarbio, 11,995) medium containing 10% fetal bovine serum (FBS, Gibco, 10,099–141) was used for cell culturing in a 5% CO2 incubator at 37°C.

### Cell transfection

Small interfering RNAs (siRNA) and plasmid vectors were transfected by using Lipofectamine 2000 (Invitrogen, 11668019), according to the manufacturer’s protocol. The sequence of siRNA was as follows: si-LINC01234-1, sense: 5’-GGCAUUAAGCCAGAUUGAGUCUUAA-3’, antisense: 5’-UUAAGACUCAAUCUGGCUUAAUGCC-3’; si-LINC01234-2, sense: 5’-AGUUGAACCAAUCACUGUGCAUUUG-3’, antisense: 5’-CAAAUGCACAGUGAUUGGUUAACU-3’. Human LINC01234 short hairpin RNA (shRNA) targeting LINC01234 was transfected as lentivirus. Cells were collected for qRT-PCR analysis after transfection for 48 hours.

### CCK-8 assay

CCK-8 assay was performed using 96-well plates to seed cells with 3 × 10^3^ per well and six replicates were performed in each group. Relative cell growth was detected using CCK-8 (Cell Counting Kit-8, Dojindo, Kumamoto, Japan) every 24 hours, according to the manufacturer’s instructions.

### Colony formation assay

Colony formation assay was performed using 6-well plates to seed cells with 1 × 10^3^ per well and three replicates were performed in each group. Cells were maintained for about 14 days. Cell culture was terminated by fixing with 4% paraformaldehyde and staining with 0.1% crystal violet for 30 minutes, respectively. The numbers of the stained colony were counted to determine the colony formation.

### Flow cytometric analysis

The protocol for the flow cytometric assay was performed as previously described [16]. Harvested cells transfecting for 48 hours were analyzed by flow cytometer (BD Biosciences) after propidium iodide (PI) staining. The Flowjo10 software was used to count and compare the percentages of the cells in the G0/G1, S, and G2/M phases.

### Animal model construction

All protocols involving animals were performed in strict accordance with the recommendations in the Guide for the Care and Use of Laboratory Animals of the NIH (Bethesda, MD) and approved by the ethics committee of the Ruijin Hospital, Shanghai Jiao Tong University School of Medicine. One side of the armpit regions of the male BALB/c nude mice (6–8 weeks old) was subcutaneously injected with 1 × 10^6^ cells. Tumor volumes were measured every seven days. The subcutaneous tumors were harvested after four weeks after injection. The harvested tumor tissues were sliced and subjected to immunohistochemistry (IHC) staining [17].

### Western blot

Total protein was extracted using RIPA solution. SDS-PAGE (10%) gel and nitrocellulose filter membrane (0.22 mm) were used to separate and transfer protein. The primary antibodies used were as follows: Cyclin D1 (CST, #2922, 1: 1000), p53 (Abcam, ab32389, 1: 1000), p21 (Abcam, ab109520, 1: 2000), BRD4 (Proteintech, 67374-2-Ig, 1: 5000). GAPDH antibody was used as a control.

### RNA immunoprecipitation

RNA immunoprecipitation (RIP) was used to investigate whether LINC01234 and miR-140-3p could interact or bind with the potential binding protein Ago2 in ACC cells. An EZMagna RIP kit (Millipore-17-701) was used according to the manufacturer’s instructions and the immunoprecipitated RNA was subjected to qRT-PCR to analyze LINC01234 content.

### Dual-Luciferase reporter assay

Dual-Luciferase Reporter Assay was implemented as previously described [16]. The complementary DNA fragment containing the wild-type or mutant LINC01234 fragment and the 3’-untranslated region (3’-UTR) of BRD4 was subcloned downstream of the luciferase gene within the pGL3-basic luciferase reporter vector (Promega). These plasmids were co-transfected into ACC cells together with the miR-140-3p mimic. The Dual-Luciferase Reporter Assay kit (Promega, E1910, USA) was used to consecutively measure the firefly and *Renilla* luciferase activities in cell lysates after transfection for 48 hours.

### Statistical analysis

Data were shown as mean ± SD. Data analysis was conducted using the GraphPad Prism 5 software. A P value of < 0.05 was considered statistically significant. All tests were two-sided.

## Results

In this study, by comparing pathological-associated lncRNA expressions in GSE61359 tumors and normal controls, LINC01234 was selected to further investigate its role in ACC. Data mining revealed that the significantly up-regulated LINC01234 expression was observed in ACC compared with that in control patients. And a shorter survival time presents in patients with higher LINC01234 expression compared to that in patients with lower LINC01234 expression. LINC01234 silencing resulted in cell growth arrest in vitro and in vivo. Mechanism studies suggested that LINC01234 silencing induced cell cycle arrest, and that BRD4 overexpression could restore these phenomena. Further research showed that LINC01234 could mediate BRD4 expression through competitively sequestering miR-140-3p, as evidenced by the positive correlation of LINC01234 with BRD4 and the inverse correlation with miR-140-3p expression. Luciferase activity assay also verified the targeting relationship between LINC01234, BRD4, and miR-140-3p. Up-regulated LINC01234 in ACC cells significantly reversed the degradation of BRD4 by miR-140-3p.

### Identification of pathological stage-associated modules and functional enrichment analysis

After preliminary data processing, a total of 14,334 AEGs were obtained after genes with low expression were removed. The average linkage method combined with the Pearson correlation method was used to perform sample clustering. Then, 17 outlier samples were removed, and the remaining 62 samples were saved for subsequent analysis (Figure 1a). When soft-thresholding power β was set to 10, the constructed network was in accordance with the characteristics of the scale-free network (R^2^ > 0.9) (Figure 1b, c). We identified 25 co-expressed modules (Figure 1d) after average linkage hierarchical clustering of the AEGs.

**Figure 1.** Sample clustering analysis and module trait heatmaps are shown. (a) Sample dendrogram and trait map of patients with adrenocortical carcinoma (survival time, survival status, pathological stage, and Weiss score) (b) Different soft-thresholding powers β (x-axis) for different scale-free fit indexes (y-axis) (c) Different soft-thresholding powers (x-axis) for different mean connectivity (y-axis) (d) Cluster dendrogram of the lncRNAs and mRNAs (e) Heatmap displaying the relationship between clustered modules and the pathological stage of patients with adrenocortical carcinoma. Weiss score: white represents the lowest score, red represents the highest score, and the darker the color, the higher the score, overall survival (OS): White represents survival and red represents death; OS time: the closer to red, the shorter the time; stage: the closer to red, the higher the stage.

Next, by performing correlation analysis between modules and pathological stages, we found that the greenyellow, blue, and lightsteelblue modules exhibited a higher module significance (MS) with the pathological stage (MS of the greenyellow module = 0.54 and MS of the lightsteelblue module = 0.52) (Figure 1e). This result suggests that genes in the two modules are strongly associated with the pathological stage of patients with ACC.

### Up-regulated LINC01234 indicated a poor prognosis in patients with ACC

Greenyellow and lightsteelblue modules, which had a higher MS among the 25 co-expression modules, were analyzed to identify potential dysregulated lncRNAs that may have participated in ACC progression. In these two modules, 75 lncRNAs were selected; among them, 44 were detected in the GSE61359 dataset. Significantly up-regulated or down-regulated lncRNAs were present in tumor (containing ACC and ACA) tissues in contrast with a normal adrenal cortex (Figure 2a). Notably, LINC01234 had a higher log2 (fold change) in ACC vs normal tissue (Figure 2b) than in ACA vs normal tissue (Figure 2c). The detail expression changes of LINC01234 in GSE61359 are shown in Figure 2d. Concurrently, another GEO dataset (Figure 2e, GSE33371) was used to analyze the expression pattern of LINC01234 in ACC. Moreover, the GSE33371 dataset shows that a higher LINC01234 expression implied larger tumor volume when the average value of LINC01234 expression was taken as the cutoff. The relationship between the patients’ ACC prognosis and LINC01234 expression level was then evaluated. For this analysis, the median expression level of LINC01234 expression was taken as the cutoff. Using the GEPIA database, the results showed that shorter overall survival (OS) (Figure 2f) and disease-free survival (DFS) (Figure 2g) times existed in patients with higher LINC01234 levels. Collectively, the data above suggested that LINC01234 exerts cancer promoting factors in ACC.

**Figure 2.** Up-regulated LINC01234 expression in ACC indicated a poor prognosis by TCGA-ACC data mining. (a–c) Volcano plot showing fold changes (log2, x-axis) of lncRNAs and corresponding p-values (−log10, y-axis) of all cancer tissue (ACA and ACC) vs normal tissue, ACC vs normal tissue, and ACA vs normal tissue in GSE61359. Log2 fold change values >1 are represented by a red dot and log2 fold change values <1 are represented by a blue dot (student’s t-test). (d and e) LINC01234 expression was analyzed in ACC, ACA, and normal tissues using GSE61359 and GSE33371. (***p < 0.001) (f) Kaplan–Meier analysis of the overall survival rate according to LINC01234 expression levels in TCGA-ACC (p = 0.037) (g) Kaplan–Meier analysis of the disease-free survival rate according to LINC01234 expression levels in TCGA-ACC cohort (p = 0.035).

### Down-regulated LINC01234-inhibited ACC cancer cell growth

In order to study the biological functions of LINC01234 in ACC, siRNA was transfected into SW-13 and H295R cells to knockdown LINC01234 (Figure 3a). Using CCK-8 assays, we found that LINC01234 silencing significantly slowed SW-13 (Figure 3b) and H295R (Figure 3c) cell proliferation. Likewise, through colony formation assays, we found that the clonogenic survival of SW-13 (Figure 3d,e) and H295R (Figure 3f,g) cells was markedly inhibited by LINC01234 down-regulation. Following these procedures, shRNA of LINC01234 or control vector were stably transfected into SW-13 cells to detect the effects of LINC01234 on tumor growth *in vivo*. Subcutaneous tumor formation (Figure 3h) revealed that the group injected with sh-LINC01234 cells possessed a significantly smaller average size (Figure 3i) and weight (Figure 3j) of tumors than the control. Finally, IHC staining revealed a weaker Ki-67 proliferation marker existed in sh-LINC01234 tumors than in control groups (Figure 3k). In summary, these results verified the carcinogenic role of LINC01234 in ACC.

**Figure 3.** The effects of LINC01234 on ACC cell proliferation *in vitro* and *in vivo* are shown. (a) The qRT-PCR method was performed to analyze LINC01234 expression in NC-, si-LINC01234-1-, and si-LINC01234-2-treated ACC cells. (b and c) The viability of NC-, si-LINC01234-1-, and si-LINC01234-2-transfected ACC cells was determined by CCK-8 assays. (d–g) The proliferation of NC-, si-LINC01234-1-, and si-LINC01234-2-transfected ACC cells was determined by colony formation assays. (h) The stable LINC01234 knockdown in SW-13 cells inhibited tumor formation *in vivo*. (i) Tumor volume curves showed that tumor growth rate was slowed when treated with stable LINC01234 knockdown in SW-13 cells. (j) Tumor weights were shown in two groups. (k) Ki-67 levels existed in tumor tissues from sh-LINC01234 or control SW-13 cells. NC = negative control, the data shows as mean ± SD. (*p < 0.05, **p < 0.01, ***p < 0.001).

### LINC01234 regulates cell cycles in ACC

To clarify the molecular mechanism of LINC01234 participation in ACC, we performed gene set enrichment analysis (GSEA). The results revealed that the cell cycle was positively related to a higher LINC01234 expression (Figure 4a). Hence, we conducted PI assay to analyze the change of cell cycles with or without LINC01234 knockdown. The results revealed that the elevated ratio of G0/G1 was displayed after LINC01234 knockdown in SW-13 (Figure 4b) and H295R (Figure 4c) cells. Meanwhile, cell cycle-related genes, including down-regulated Cyclin D1, up-regulated p53, and p21, were observed in ACC cells after LINC01234 knockdown (Figure 4d), indicating that LINC01234 participates in regulating cell cycles.

**Figure 4.** LINC01234 is involved in the regulation of cell cycles in ACC. (a) The bubble diagram shows the associated signaling pathway results from gene enrichment analysis based on the LINC01234 expression using TCGA-ACC dataset. NES stands for normalized enrichment score. (b and c) The cell cycle was arrested in SW-13 and H295R cells after LINC01234 knockdown. The bar chart represents the percentage of cells in the G0/G1, S, and G2/M phases, respectively. (d) Expressions of CyclinD1, p53, and p21 were detected after LINC01234 knockdown.

### LINC01234 participates in the cell cycle regulation via mediating BRD4 expression

GSEA results revealed that folate biosynthesis was closely related to LINC01234 expression (Figure 4a). Folate cycle-related gene analysis showed that BRD4 expression was related to pathological stage (Figure 5a). The detail expression changes in GSE61359 showed that significantly up-regulated BRD4 was present in ACC and ACA tissues in contrast with a normal adrenal cortex (Figure 5b). Using the GEPIA database, we evaluated the relationship between the patients’ prognosis and the BRD4 expression level. For this analysis, the median expression level of BRD4 expression was taken as the cutoff. The results showed that shorter OS (Figure 5c) and DFS (Figure 5d) times existed in patients with higher BRD4 levels. Moreover, a positive relationship between LINC01234 expression and BRD4 expression was presented using Pearson correlation analysis (Figure 5e). BRD4 expression was decreased after LINC01234 knockdown (Figure 5f). Cell cycle assays revealed restored cell cycle arrest after BRD4 overexpression in LINC01234 knockdown cells (Figure 5g,h). Herein, we concluded that LINC01234 regulated cell cycles in ACC by mediating BRD4 expression.

**Figure 5.** LINC01234 participates in the cell cycle regulation via mediate BRD4 expression. (a) Online analysis of GEPIA revealed that BRD4 expression was related to pathological stage. (p = 0.0104) (b) BRD4 expression was analyzed in ACC, ACA, and normal tissues using GSE61359. (*p < 0.05, **p < 0.01) (B) BRD4 expression was analyzed in ACC, ACA, and normal tissues using GSE61359. (*p < 0.05, **p < 0.01) (c) Kaplan–Meier analysis of the overall survival rate according to BRD4 expression levels in TCGA-ACC (p = 0.066) (d) Kaplan–Meier analysis of the disease-free survival rate according to BRD4 expression levels in TCGA-ACC cohort (p = 3.9e−05) (e) A positive relationship between LINC01234 expression and BRD4 expression was revealed by Pearson correlation analysis through an online analysis of GEPIA. (r = 0.43, p < 0.001) (f) Expressions of BRD4 were detected after LINC01234 knockdown. (g and h) Cell cycle arrest by LINC01234 knockdown was partially restored after BRD4 overexpression in SW-13 and H295R cells.

### MiR-140-3p may mediate a ceRNA network with LINC01234 and BRD4

Accumulating evidence has shown that lncRNAs are acting as competing endogenous RNAs (ceRNAs) for miRNAs to allow expression of targeted genes [18]. Hence, to investigate the molecular link between LINC01234 and BRD4, which forms a ceRNA network, online bioinformatic databases were used. As shown in Figure 6a, 332 miRNAs were predicted to bind to the LINC01234 sequence (the threshold is 0.7) using the LncBase Predicted v.2 DIANA tool (www.microrna.gr/LncBase) with parameters set according to the website without any adjustment. Additionally, DIANA’s TarBase v8.0 tool (http://www.microrna.gr/tarbase) with parameters set according to the website without any adjustment, showed that 120 miRNAs experimentally supported interaction with BRD4. Meanwhile, 227 miRNAs were predicted to target BRD4 according to the starBase v2.0 software (ENCORI) (http://starbase.sysu.edu.cn/) with parameters set according to the website without any adjustment. Among them, miR-140-3p (has-miR-140-3p) was the only overlapped miRNA in the above three intersections (Figure 6a). Next, we found that both the expression of BRD4 (Figure 6b) and LINC01234 (Figure 6c) were negatively associated with the expression of miR-140-3p in TCGA-ACC dataset analyzed by starBase v2.0. Furthermore, down-regulated miR-140-3p expression often indicated a poor prognosis of ACC (Figure 6d, p = 0.033). Therefore, miR-140-3p was chosen as a candidate for further investigation.

**Figure 6.** MiR-140-3p may be involved in a ceRNA network with LINC01234 and BRD4. (a) The number of predicted miRNA sponging by LINC01234 is 332 according to the LncBase Predicted v.2 tool (DIANA). The number of experimentally validated miRNAs targeting BRD4 is 120 and 227, according to the TarBase v8.0 tool (DIANA) and the starBase v2.0 software (ENCORI), respectively. The overlapped miRNAs in the above three intersections are hsa-miR-140-3p. (b) Association analysis of the relationship between miR-140-3p and BRD4 expression levels was revealed by online analysis using starBase v2.0. (r = −0.308, p = 5.83e−03) (c) Association analysis of the relationship between miR-140-3p and LINC01234 expression levels was revealed by online analysis using starBase v2.0. (r = −0.354, p = 1.36e−03) (d) Kaplan–Meier analysis of the overall survival rate according to miR-140-3p expression levels was revealed by online analysis using starBase v2.0. (p = 0.033).

### LINC01234 mediates BRD4 expression by competitively binding miR-140-3p in ACC

To confirm the potential interaction between LINC01234 and miR-140-3p, a sequence of mutations was made in the miR-140-3p binding site of LINC01234 (mut-LINC01234, (Figure 7a), the wild type referred to as wt-LINC01234). Dual-Luciferase Reporter Assay showed that miR-140-3p-mediated inhibition of luciferase activity was abolished in the mut-LINC01234 group compared with that in the wt-LINC01234 group (Figure 7b) and the levels of miR-140-3p were increased significantly after LINC01234 knockdown (Figure 7c). Additionally, RIP experiments showed that LINC01234 and miR-140-3p were enriched in immunoprecipitated Ago2 compared with that in the control IgG (Figure 7d).

**Figure 7.** BRD4 is targeted by miR-140-3p, which forms a spongy body with LINC01234. (a) The binding sites between LINC01234 and miR-140-3p were predicted using starBase v2.0. LINC01234 mutated at the putative binding site. (b) Dual-Luciferase Reporter Assay was performed to verify that miR-140-3p was binding with LINC01234 in ACC cells. (c) MiR-140-3p expression was measured in LINC01234 knockdown ACC cells using qRT-PCR. (d) RIP experiments were performed in ACC cells to detect the binding between LINC01234 and Ago2 or its matching IgG control. (e) Schematic view of the binding sites of miR-140-3p in the wild-type (WT) or mutant (Mut) 3’-UTR region of BRD4 is shown. (f) The luciferase reporte*r plasmid* containing WT and Mut BRD4 was co-transfected into ACC cells with miR-140-3p or corresponding empty plasmid vector. (g) BRD4 expression was measured in ACC cells transfected with miR-140-3p mimics, miR-140-3p inhibitors, or corresponding control miRNAs using qRT-PCR. (h-j) Relative protein levels of BRD4 were measured in ACC cells transfected with miR-140-3p mimics (h), miR-140-3p inhibitor (i), or corresponding control miRNAs (j). BRD4 protein level in ACC cells following knockdown of LINC01234 and/or miR-140-3p mimics is shown. The data shows as mean ± SD. (*p < 0.05, **p < 0.01, ***p < 0.001).

Subsequently, to verify the interaction between miR-140-3p and BRD4, the putative binding site between miR-140-3p and the 3’-UTR of BRD4 was determined using starBase v2.0 (Figure 7e). Dual-luciferase reporter assay showed that miR-140-3p significantly decreased the luciferase activity of report genes containing wild-type BRD4 (wt-BRD4), while there was no effect on the mutated 3’-UTR BRD4 (mut-BRD4) in ACC cells (figure 7f). Moreover, we overexpressed miR-140-3p and found that the levels of BRD4 were significantly decreased, whereas miR-140-3p knockdown displayed an opposite effect (Figure 7g); a similar phenomenon occurs at protein levels (Figure 7h,i). In light of the fact that LINC01234 can sponge miR-140-3p, we examined whether miR-140-3p plays a role in the relationship between LINC01234 and BRD4. The results showed that sh-LINC01234-mediated down-regulation of BRD4 was effectively reversed by miR-140-3p inhibitors (Figure 7j). Collectively, the data above suggested that LINC01234 modulates BRD4 expression by competitively binding miR-140-3p.

## Discussion

In ACC, initial staging is the most important factor in determining prognosis. In the early stage, the five-year survival rate of patients with ACC could be up to 80% [1–3]. However, most patients in this study were diagnosed at an advanced stage and the five-year survival rate was less than 15%, with a high recurrence rate even after radical surgery [8]. Hence, it is necessary to explore novel biomarkers for patients with ACC to predict the pathological stage and prognosis in an accurate and timely manner. WGCNA is a novel gene screening method that can be used to explore relationships between pathological traits and expression profiles [5]. Previously, WGCNA has revealed abundant potential biomarkers for the prognostic prediction of tumors [19,20]. For example, CDCA5, ANLN, ASPM, KIAA0101, CENPF, FOXM1, PRC1, RACGAP1, TPX2, MELK, NDC80, and SPAG5 were predicted by WGCNA to be related to the tumor grade and prognosis in ACC [21]. Hence, WGCNA was used to predict pathological stage-associated genes, including lncRNAs.

LncRNA co-expression analysis has been performed in multiple cancer cases to identify prognostic lncRNA biomarkers, but no corresponding similarity analysis has been performed in ACC [7,22]. In this study, we constructed 25 co-expression modules related to the clinical traits of patients with ACC by using the WGCNA R package [5]. And pathological-associated LINCRNAs was selected. Subsequent analysis revealed that LINC01234 had the highest fold change with statistical significance, and larger tumor sizes and shorter outcome times were correlated with a higher expression of LINC01234 in patients with ACC. Assays indicated that LINC01234 silencing inhibited cell growth *in vitro* and *in vivo*. These results suggest that LINC01234 is carcinogenic and can be considered as a potential prognostic indicator for ACC, which is similar to the biological function previously reported in other tumors [15,16].

The GSEA analysis showed that a high LINC01234 expression was positively correlated with cell cycles in ACC. Meanwhile, flow cytometric analysis confirmed the role of LINC01234 on cell cycle regulation in ACC cells, and the protein expression level of cell cycle-related markers, including Cyclin D1, p53, and p21, was also confirmed [23]. As it is known, the key checkpoint protein Cyclin D1 is responsible for cell cycle transformation from the S phase to the G1 phase via participation in transcriptional regulation and DNA repair [24]. Additionally, p53 and p21 can regulate cell cycles in many ways, including DNA repair and transcriptional regulation [25,26]. Inspired by this, we speculated that LINC01234 may be involved in DNA repair or transcriptional regulation to regulate cell cycles; further evidence should be collected to verify this.

The GSEA analysis also revealed that a high LINC01234 expression was positively related to folate biosynthesis. Folate, through its key role in C1 metabolism, is essential for DNA repair and synthesis, as well as DNA methylation [27,28]. This gives us more reason to suspect that LINC01234 may be involved in DNA repair. The relationship between LINC01234 and folate cycle-related genes was then analyzed. We found that BRD4, which interacts with the folate pathway key enzyme MTHFD1 to link folate metabolism to transcriptional regulation [29], was positively related to LINC01234. BRD4, acting as a histone acetyl-reader, is an important regulator of chromatin structure, which plays a role in cancer progression, cell proliferation, DNA damage, and gene regulation [30]. Previous studies have determined that MTHFD1L silencing is related to cell cycle delay [31]. The result above revealed that BRD4 overexpression could restore cell cycle arrest resulting from LINC01234 knockdown. Therefore, we speculated that LINC01234 may affect the cell cycles in ACC by affecting the binding of BRD4 and MTHFD1L.

Generally, lncRNAs exert function by absorbing miRNA sponges and they play a role in ceRNAs. Several LINC01234–miRNA–mRNA trios have been identified as the main mechanisms promoting tumorigenesis. For example, in gastric cancer, LINC01234 functions as an miR-204-5p sponge to up-regulate the expression of CBFB [16]. In HCC, LINC01234 was reported to be implicated in resistance to chemotherapy via the miR-31-5p/MAGEA3 axis [14]. As it is known, the miRNA target is the core component of the ceRNA network. Inspired by this, we speculated that LINC01234 may also play a role in ceRNAs in connection with post-transcriptional regulation of BRD4 and miRNAs in ACC. To determine this hypothesis, bioinformatic analysis and luciferase reporter assays were conducted to confirm that miR-140-3p possesses the putative binding site of LINC01234 and BRD4. Furthermore, RNA-IP assay showed that LINC01234 was significantly pulled down in miR-140-3p overexpressing cells and the miR-140-3p inhibitor could effectively reverse the down-regulation of BRD4 mediated by sh-LINC01234. Thus, these results indicated that BRD4 is a downstream target of LINC01234 by sponging miR-140-3p in ACC cells. Previous studies confirmed that miR-140-3p worked as a tumor suppressor in various kinds of cancer [32,33]. Therefore, more studies should be conducted to explore the role of miR-140-3p exertion in ACC. In addition, LINC01234 was reported to work through miR-204-5p [16], miR-31-5p [14], etc. Therefore, LINC01234 may partly function through sponging miR-140-3p in ACC. As a further matter, other miRNAs may also be target regulated by LINC01234 in ACC. Hence, further study needs to be conducted to discover potential miRNAs.

In summary, we determined for the first time that pathological stage-associated lncRNA LINC01234 was overexpressed in ACC, and it is a prognostic risk factor in ACC. LINC01234 plays a carcinogenic role via regulating cell cycles in ACC through the miR-140-3p/BRD4 axis. A better understanding of LINC01234 in ACC development was provided in the current study. LINC01234 has the potential to be a novel target in ACC management.

## Conclusion

In conclusion, LINC01234 was proved to functions as a ceRNA to regulate BRD4 expression by sponging miR-140-3p in ACC progress. And higher LINC01234 expression observed in ACC patients indicated worse prognosis, which may be a useful candidate for ACC diagnosis and therapy.

## Supplementary Material

Supplemental Material
